The article "Activation of endoplasmic reticulum stress promotes autophagy and apoptosis and reverses chemoresistance of human small cell lung cancer cells by inhibiting the PI3K/AKT/mTOR signaling pathway" was retracted in 2019. Reasons: errors in the analysis; false authorship; concerns about the results or conclusions; concerns about a third party's involvement.

# Activation of endoplasmic reticulum stress promotes autophagy and apoptosis and reverses chemoresistance of human small cell lung cancer cells by inhibiting the PI3K/AKT/mTOR signaling pathway

**DOI:** 10.18632/oncotarget.12718

**Published:** 2016-10-18

**Authors:** Xin-Shuang Yu, Juan Du, Yu-Jun Fan, Feng-Jun Liu, Li-Li Cao, Ning Liang, De-Guo Xu, Jian-Dong Zhang

**Affiliations:** ^1^ Department of Radiation Oncology, Shandong Provincial Qianfoshan Hospital, Shandong University, Jinan 250014, P.R. China; ^2^ Medical Research Center, Shandong Provincial Qianfoshan Hospital, Shandong University, Jinan 250014, P.R. China; ^3^ Medical Management Service Center of Shandong Provincial Health and Family Planning Commission, Jinan 250014, P.R. China

**Keywords:** endoplasmic reticulum stress, PI3K/AKT/mTOR signaling pathway, small cell lung cancer, autophagy, apoptosis

## Abstract

**Objective:**

This study aims to investigate the effects of endoplasmic reticulum stress (ERS) on autophagy, apoptosis and chemoresistance of human small cell lung cancer (SCLC) cells via the PI3K/AKT/mTOR signaling pathway.

**Results:**

The expressions of ERS-related proteins (PEAK, eIF2α and CHOP) up-regulated, autophagy-related proteins (LC3, LC3-II and Beclin1) and apoptosis-related proteins (Bax and procaspase-3) down-regulated in NCI-H446 and H69 cells after tunicamycin treatment for 24 h. Compared with the blank group, the tunicamycin, BEZ235 and tunicamycin + BEZ235 groups exhibited decreased expressions of p-PI3K, p-AKT and p-mTOR, and increased expressions of autophagy-related proteins (LC3, LC3-II and Beclin1) and apoptosis proteins (Bax and procaspase-3), and the most obvious changes were observed in the tunicamycin + BEZ235 group.

**Materials and Methods:**

CCK-8 assay was applied to select the best cell line from five SCLC cell lines (NCI-H446, H69, H526, H146 and H209). Finally, NCI-H446 and H69 cells were selected for further experiments. NCI-H446/CDDP and H69/CDDP were selected and divided into the blank group, tunicamycin (an ESR inducer) group, BEZ235 (inhibitors of PI3K/AKT/mTOR pathway) group and tunicamycin + BEZ235 group. Cell apoptosis was detected by flow cytometry. Autophagy was observed by fluorescence microscopy and flow cytometry. Western blotting was used to detect the expressions of ERS-related proteins, autophagy-related proteins, apoptosis-related proteins and PI3K/AKT/mTOR pathway-related proteins.

**Conclusions:**

Our findings provide evidence that the activation of ERS could promote autophagy and apoptosis and reverse chemoresistance of human SCLC cells by inhibiting the PI3K/AKT/mTOR pathway.

## INTRODUCTION

As a highly malignant pulmonary neuroendocrine tumor, small-cell lung cancer (SCLC) represents 15% of all lung cancer with a high proliferative index and a strong possibility of early metastasis [1]. The prognosis of SCLC remains notably poor and therapeutic development has lagged behind non-small cell lung cancer (NSCLC) [2]. About two-thirds of SCLC patients were diagnosed in advanced stage with metastases in the lung, liver and brain with an overall survival of SCLC at 5 years being 5–10% [3]. Despite a high sensitivity to the initial chemotherapy and radiotherapy, the 2-year survival rate of patients with limited disease SCLC is about 25%, and the survival rate continues to decrease after 2 years [4, 5]. As a particularly aggressive form of lung cancer, SCLC is characterized by early metastasis, with the ability to develop resistance against chemotherapeutic drugs [6].

The article "Activation of endoplasmic reticulum stress promotes autophagy and apoptosis and reverses chemoresistance of human small cell lung cancer cells by inhibiting the PI3K/AKT/mTOR signaling pathway" was retracted in 2019. Reasons: errors in the analysis; false authorship; concerns about the results or conclusions; concerns about a third party's involvement.

Endoplasmic reticulum (ER) is a major organelle having many cellular functions and is an essential site for maintaining homeostasis [7]. When ER related pathways of protein folding regulation, post-translational modifications, cellular metabolism and calcium signaling are disturbed, the accumulation of misfolded proteins within the ER might ultimately leads to ER stress (ERS) [8]. With overwhelmed ERS, cells initiate autophagy, which is followed by large-scale degradation and apoptosis [9]. Autophagy is an evolutionarily conserved intracellular process, by which bulk cytoplasm is enveloped in a double-membrane vesicle and shuttled to lysosomes for degradation, participating in stress tolerance [10, 11]. Autophagy is demonstrated to be ectopically activated in tumor cells, which confers to chemoresistance [12–14]. ERS might promote autophagy by releasing calcium to activate calcium-dependent kinase kinase-βand adenosine monophosphate-activated protein kinase, and inhibit mammalian target of rapamycin (mTOR) [15]. Activating ERS has attracted a great deal of attention for cancer therapy due to the fact that ERS can effectively enhance tumor cell apoptosis [16]. ERS can decrease cisplatin sensitivity to ovarian carcinoma cells by regulating cell autophagy via the pathways of mTOR and Beclin1 [17]. Chen et al. demonstrated that cxc195 and ERS induced apoptosis, inhibited phosphoinositide 3-kinase (PI3K)/AKT/mTOR signaling pathway in HepG2 cells [18]. In the present study, we aimed investigate the effects of ERS on autophagy, apoptosis and chemoresistance of human SCLC cells via the PI3K/AKT/mTOR signaling pathway, in order to provide a new therapeutic direction for SCLC patients.

## RESULTS

### Effects of different doses of tunicamycin on the viability of SCLC cells

After 24 h of tunicamycin (5 ug/mL), cell viabilities of five SCLC cell lines were shown in Figure 1A. The viability of NCI-H446and H69 cells were obviously higher than that of H526, H146and H209 cells (all *P* < 0.05) (Figure 1A). Therefore, NCI-H446 and H69 cells were selected for further experiments.

The article "Activation of endoplasmic reticulum stress promotes autophagy and apoptosis and reverses chemoresistance of human small cell lung cancer cells by inhibiting the PI3K/AKT/mTOR signaling pathway" was retracted in 2019. Reasons: errors in the analysis; false authorship; concerns about the results or conclusions; concerns about a third party's involvement.

**Figure 1:** Effects of different doses of tunicamycin on the viability of human small cell lung cancer (SCLC) cells (**A**) comparison of the viability of five SCLC cell lines treated with 5 ug/mL tunicamycin for 24 h; *stands for *P* < 0.05 in comparison with NCI-H446 cells; ^#^stands for *P* < 0.05 in comparison with H69 cells; (**B**) changes in NCI-H466 cell viability after treated with different doses of tunicamycin; (**C**), changes in H69 cell viability after treated with different doses of tunicamycin; *stands for *P* < 0.05 in comparison with 0 ug/mL tunicamycin.

The effects of tunicamycin on the viability of NCI-H446 and H69 cells were in a dose-dependent and time-dependent manner. With the increasing doses of tunicamycin, the effects of the tunicamycin on the viability of NCI-H446 and H69 cells were increased continuously (all *P* < 0.05) (Figure 1B and 1C). The IC50 values after 24 h of tunicamycin treatment on NCI-H446 and H69 cells were 3.01 ± 0.14 μg/mL and 2.94 ± 0.16 μg/mL, respectively.

### Effects of different doses of tunicamycin on the expressions of ESR-related proteins and PI3K/AKT/mTOR signaling pathway-related proteins in NCI-H446 and H69 cells

Tunicamycin can activate ERS and up-regulate the expressions of ERS-related proteins (PERK, eIF2α and CHOP) in a dose-dependent and time-dependent manner (all *P* < 0.05) (Figure 2). The tunicamycin can inhibit PI3K/AKT/mTOR signaling pathway and down-regulate the expressions of p-PI3K, p-AKT and p-mTOR, and the effects were increased significantly with the increasing doses of tunicamycin (all *P* < 0.05). However, the expressions of PI3K, AKT, or mTOR showed no changes in NCI-H446 and H69 cells at 24 after tunicamycin treatment (Figure 3). These results suggest that the activation of ERS could inhibit the PI3K/AKT/mTOR signaling pathway.

**Figure 2:** Effects of different doses of tunicamycin on the activation of endoplasmic reticulum stress (ERS) in NCI-H446 and H69 cells (**A**), ERS-related protein expressions in NCI-H446 cells after treated with different doses of tunicamycin for 24 h; (**B**), ERS-related protein expressions in H69 cells after treated with different doses of tunicamycin for 24 h; *stands for *P* < 0.05 in comparison with 0 ug/mL tunicamycin.

**Figure 3:** Effects of different doses of tunicamycin on the PI3K/AKT/mTOR signaling pathway in NCI-H446 and H69 cells (**A**), the expressions of PI3K/AKT/mTOR signaling pathway-related proteins in NCI-H446 cells after treated with different doses of tunicamycin for 24 h; (**B**), the expressions of PI3K/AKT/mTOR-related proteins in H69 cells after treated with different doses of tunicamycin for 24 h; *stands for *P* < 0.05 in comparison with 0 ug/mL tunicamycin.

The article "Activation of endoplasmic reticulum stress promotes autophagy and apoptosis and reverses chemoresistance of human small cell lung cancer cells by inhibiting the PI3K/AKT/mTOR signaling pathway" was retracted in 2019. Reasons: errors in the analysis; false authorship; concerns about the results or conclusions; concerns about a third party's involvement.

### Effects of different doses of tunicamycin on the autophagy and apoptosis of NCI-H446 and H69 cells

Tunicamycin can induce autophagy of NCI-H446 and H69 cells and regulate the expressions of autophagy-related proteins. With the increasing doses of tunicamycin, the protein expressions of LC3, LC3-II and Beclin1 increased continuously, but the protein expressions of LC3-I and p62 decreased continuously (all *P* < 0.05) (Figure 4). Also, tunicamycin can promote apoptosis of NCI-H446 and H69 cells by up-regulating the expressions of procaspase-3 and Bax, and down-regulate the expression of Bcl-2. The effects were increased significantly with increased concentrations (all *P* < 0.01) (Figure 5). These results indicate that the activation of ERS could induce autophagy and promote apoptosis of NCI-H446 and H69 cells.

**Figure 4:** Effects of different doses of tunicamycin on the autophagy of NCI-H446 and H69 cells (**A**) MDC fluorescence intensity of NCI-H446 and H69 cells after treated with different doses of tunicamycin for 24 h; (**B**) the expressions of autophagy-related proteins in NCI-H446 and H69 cells after treated with different doses of tunicamycin for 24 h; *stands for *P* < 0.05 in comparison with 0 ug/mL tunicamycin.

**Figure 5:** Effects of different doses of tunicamycin on the apoptosis of NCI-H446 and H69 cells (**A**), the apoptosis rate of NCI-H446 and H69 cells after treated with different doses of tunicamycin for 24 h; (**B**) the expressions of apoptosis-related proteins in NCI-H446 and H69 cells after treated with different doses of tunicamycin for 24 h; *stands for *P* < 0.05 in comparison with 0 ug/mL tunicamycin.

### Effects of tunicamycin and BEZ235 on the expressions of ERS-related proteins, PI3K/AKT/mTOR signaling pathway-related proteins, autophagy-related proteins and apoptosis-related proteins in NCI-H446/CDDP and H69/CDDP cells

Both BEZ235 and tunicamycin can inhibit the activation of PI3K/AKT/mTOR signaling pathway, and promote the autophagy and apoptosis of NCI-H446/CDDP and H69/CDDP cells. Compared with the blank group, at 24 h after BEZ235 and tunicamycin treatment, the expressions of the expressions of p-PI3K, p-AKT and p-mTOR were significantly decreased, while the expressions of ERS-related proteins, autophagy-related proteins and apoptosis-related proteins were obviously increased in the tunicamycin, BEZ235 and tunicamycin + BEZ235 groups (all *P* < 0.05) (Figures 6–9). Furthermore, these changes in the tunicamycin + BEZ235 group were more obvious than those in the tunicamycin and BEZ235 groups (all *P* < 0.05). Our findings indicate that the activation of ERS could inhibit PI3K/AKT/mTOR pathway and promote autophagy and apoptosis, thereby reversing chemoresistance of NCI-H446/CDDP and H69/CDDP cells.

The article "Activation of endoplasmic reticulum stress promotes autophagy and apoptosis and reverses chemoresistance of human small cell lung cancer cells by inhibiting the PI3K/AKT/mTOR signaling pathway" was retracted in 2019. Reasons: errors in the analysis; false authorship; concerns about the results or conclusions; concerns about a third party's involvement.

**Figure 6:** Effects of tunicamycin and BEZ235 on the activation of endoplasmic reticulum stress (ERS) in NCI-H446/CDDP and H69/CDDP cells (**A**) the expressions of ERS-related proteins in NCI-H446/CDDP and H69/CDDP cells after treated with 5 ug/mL of tunicamycin or/and 64 μM of BEZ235 for 24 h; (**B**) the expressions of ERS-related proteins of NCI-H446/CDDP and H69/CDDP cells after treated with 5 ug/mL of tunicamycin or/and 64 μM of BEZ235 for 24 h; *stands for *P* < 0.05 in comparison with the blank group; ^#^stands for *P* < 0.05 in comparison with the tunicamycin group; ^&^stands for *P* < 0.05 in comparison with the BEZ235 group.

**Figure 7:** Effects of tunicamycin and BEZ235 on the PI3K/AKT/mTOR signaling pathway in NCI-H446/CDDP and H69/CDDP cells (**A**), the expressions of PI3K/AKT/mTOR signaling pathway-related proteins in NCI-H446/CDDP and H69/CDDP cells after treated with 5 ug/mL of tunicamycin or/and 64 μM of BEZ235 for 24 h; (**B**) the expressions of PI3K/AKT/mTOR signaling pathway-related proteins in NCI-H446/CDDP and H69/CDDP cells after treated with 5 ug/mL of tunicamycin or/and 64 μM of BEZ235 for 24 h; *stands for *P* < 0.05 in comparison with the blank group; ^#^stands for *P* < 0.05 in comparison with the tunicamycin group; ^&^stands for *P* < 0.05 in comparison with the BEZ235 group.

**Figure 8:** Effects of tunicamycin and BEZ235 on the autophagy of NCI-H446/CDDP and H69/CDDP cells (**A**), flow cytometry of NCI-H446/CDDP and H69/CDDP cells after treated with 5 ug/mL of tunicamycin or/and 64 μM of BEZ235 for 24 h; (**B**), the expressions of autophagy-related proteins in NCI-H446/CDDP and H69/CDDP cells after treated with 5 ug/mL of tunicamycin or/and 64 μM of BEZ235 for 24 h; *stands for *P* < 0.05 in comparison with the blank group; ^#^stands for *P* < 0.05 in comparison with the tunicamycin group; ^&^stands for *P* < 0.05 in comparison with the BEZ235 group.

**Figure 9:** Effects of tunicamycin and BEZ235 on the apoptosis of NCI-H446/CDDP and H69/CDD cells (**A**) the apoptosis rate of NCI-H446/CDDP and H69/CDDP cells after treated with 5 ug/mL of tunicamycin or/and 64 μM of BEZ235 for 24 h; (**B**) the expressions of apoptosis-related proteins in NCI-H446/CDDP and H69/CDDP cells processed by BEZ235 and TM for 24 h; *stands for *P* < 0.05 in comparison with the blank group; ^#^stands for *P* < 0.05 in comparison with the tunicamycin group; ^&^stands for *P* < 0.05 in comparison with the BEZ235 group.

The article "Activation of endoplasmic reticulum stress promotes autophagy and apoptosis and reverses chemoresistance of human small cell lung cancer cells by inhibiting the PI3K/AKT/mTOR signaling pathway" was retracted in 2019. Reasons: errors in the analysis; false authorship; concerns about the results or conclusions; concerns about a third party's involvement.

## DISCUSSION

In our study, we aim to investigate whether ERS can induce autophagy and apoptosis and reverse chemoresistance of SCLC cells by inhibiting PI3K/AKT/mTOR signaling pathway. Our results showed that tunicamycin could up-regulate proteins related to ERS signaling pathway (PEAK, eIF2α and CHOP). Tunicamycin may reverse drug resistance and improve the treatment of hepatocellular carcinomas by targeting the DPAGT1/AKT/ABCG2 signaling pathway [19]. ERS is associated with cancer development and maintenance, and is a therapeutic target for cancer treatment [20]. Tunicamycin inhibited N-glycosylation biosynthetic processes to cause ERS and toxicity in normal tissues [21]. Tunicamycin might induce ERS to protect against the transient ischemic brain injury and ERS might induce mitophagy to rescue ischemic brains [22]. PERK phosphorylates eIF2α, and the phosphorylated eIF2α promotes the activating transcription factor 4 (ATF4), while the ATF4 increases ER capacity and strongly induces CHOP [23]. The activations of PERK, eIF2α and CHOP result in the up-regulation of ER protein folding capacity and ER-associated degradation [24]. PERK is required for the activation of GSK3α/β by ERS, and the inhibition of GSK3α/β is associated with attenuated atherosclerotic development and reduced hepatic steatosis [25, 26]. Phosphorylation of eIF2α is pivotal to control global rates of protein synthesis and to modulate mRNA-specific translation [27]. Excessive phosphorylation of eIF2α decreases cancer cell survivals. Thus, eIF2α is a worthy target for drug development to enhance the cytotoxic effects of established anti-neoplastic therapies by inhibiting upstream components of the mTOR signaling pathway [28]. CHOP can regulate cell apoptosis effectors such as Bcl-2 and Bim, and eventually lead to apoptosis activation of caspase-3 [29]. Thus tunicamycin might activate ERS related proteins, PERK, eIF2α and CHOP, to promote cell apoptosis and autophagy by inhibiting the PI3K/AKT/mTOR signaling pathway.

Besides, our study found that tunicamycin could down-regulate PI3K, AKT, mTOR protein phosphorylation. The PI3K/AKT/mTOR signaling pathway is a main signaling pathway to regulate cell growth, proliferation, metabolism and survival, commonly deregulated in cancer [30]. Alterations of the PI3K/AKT/mTOR signaling pathway occur at multiple levels, leading to PI3K activation and malignant transformation [31]. The PI3K signaling pathway plays a critical role in cell growth and survival [32]. Over-activation of Akt has been reported in NSCLC cell lines, and was closely related to chemoresistance, and suggested a poor prognosis for patients with early-stage NSCLC [31, 33, 34]. The mTOR is a serine/threonine protein kinase to regulate cell growth, motility and survival, and the dysregulation of mTOR signaling pathway can be observed in cancers with PI3K and AKT being upstream regulators of mTOR signaling pathway in mammalian cells [35]. PI3K/PTEN/AKT/mTOR signaling pathway genetic variants may predict platinum-based chemotherapy response in patients with advanced NSCLC [36]. Our findings revealed that tunicamycin can inhibit cell viability of human SCLC NCI-H446 and H69 cells, activate ERS, inhibit PI3K/AKT/mTOR signaling pathway, and thus lead to autophagy and apoptosis. Liang et al. have also reported that ER stress could negatively regulate AKT/TSC/mTOR signaling pathway to enhance autophagy, which confirmed the result of the present study [37].

The article "Activation of endoplasmic reticulum stress promotes autophagy and apoptosis and reverses chemoresistance of human small cell lung cancer cells by inhibiting the PI3K/AKT/mTOR signaling pathway" was retracted in 2019. Reasons: errors in the analysis; false authorship; concerns about the results or conclusions; concerns about a third party's involvement.

In our study, the results demonstrated that the PI3K/AKT/mTOR inhibitor BEZ235 can promote autophagy and apoptosis via inhibiting PI3K/AKT/mTOR signaling pathway, thereby reversing chemoresistance. Cisplatin is a commonly used chemotherapeutic drug, but high doses of cisplatin can cause toxic effects, such as ototoxicity and nephrotoxicity [38]. Cisplatin is cross-linked with DNAs and inhibits DNA replication and transcription [39]. Once DNA is damaged, cell cycle check points were activated, which led to the delay of the cell cycle progression, either repairing or permanently eliminating the cells through inducing cell death [40]. How the cells response to cisplatin-induced DNA damage will then decide the fate of a cell, to live or die [41]. Pabla et al. demonstrated that cisplatin could induce ERS, activate apoptotic pathways and result in Caspase-dependent or -independent apoptosis [42]. AKT regulates multiple downstream targets, resulting in cell growth, survival and cisplatin resistance [43]. Cisplatin-induced DNA damage was demonstrated to cause phosphorylation of BAD at ser136 via AKT [44]. BAD is basically phosphorylated in cells with cisplatin-induced DNA damage, and the BAD phosphorylation is needed for cell viability after cisplatin treatment [40]. Cisplatin was reported to activate PI3K/AKT signaling and lead to cisplatin resistance in ovarian cancer [45]. Qin L et al demonstrated that cisplatin could induce protective autophagy, which resulted in the decrease of sensitivity to chemotherapy [46]. Due to its effectiveness and low side effects, BEZ235 is a very promising inhibitor of the PI3K/AKT signaling pathway and thus eliminates the feedback activation of PI3K activity due to mTOR inhibition [47]. It has been found that NVP-BEZ235 can inhibit gefitinib-resistant tumor proliferation by down-regulating the phosphorylation of PI3K/AKT/mTOR signaling pathway [48].

The article "Activation of endoplasmic reticulum stress promotes autophagy and apoptosis and reverses chemoresistance of human small cell lung cancer cells by inhibiting the PI3K/AKT/mTOR signaling pathway" was retracted in 2019. Reasons: errors in the analysis; false authorship; concerns about the results or conclusions; concerns about a third party's involvement.

The results of our study also showed that tunicamycin can down-regulate proteins related to autophagy, including LC3, LC3-II and Beclin1. As an autophagosomal orthologue of yeast autophagy-related genes, LC3 including LC3-I and LC3-II, plays an essential role in autophagosome formation. LC3-II is particular a specific marker of the autophagic process as it directly correlates with the number of autophagosomes [49]. Additionally, Beclin-1 is a crucial modifier of the autophagic process and has been implicated in tumor development, including ovarian, breast and prostate tumors in humans [50]. CHOP could reduce LC3-II conversion and beclin-1 expression [51]. Therefore, in the study, tunicamycin could up-regulate CHOP, according to which the expressions of LC3-II and beclin-1 were decreased.

In conclusion, our findings provide evidence that the activation of ERS could induce autophagy and apoptosis and reverse chemoresistance of human SCLC cells by inhibiting the PI3K/AKT/mTOR pathway. Our study can provide valuable clinical advices for the chemotherapy of SCLC. There are limitations, however, that we cannot deny. Due to limited funds and time, our experiment may be not deep enough. If conditions permit, we would explore the related mechanisms behind the effects of ERS on the toxicity, apoptosis after autophagy and chemotherapy resistance of SCLC cells.

## MATERIALS AND METHODS

### Cell culture and grouping

Human SCLC cell lines (NCI-H446, H69, H526, H146 and H209) were purchased from Shanghai Institute of Cell Biology, Chinese Academy of Science. The cells were cultured in a DMEM medium (Gibco Company, Grand Island, NY, USA) containing 10% fetal bovine serum (FBS) (Zhejiang Tianhang Biotechnology Co., Ltd., Hangzhou, China) and 1% of 100 U/L penicillin and 100 mg/L streptomycin (Gibco, USA). Then, CCK-8 assay was applied to select the best cell line from these five SCLC cell lines (NCI-H446, H69, H526, H146 and H209). Finally, NCI-H446 and H69 cells were selected for further experiments.

Cisplatin (CDDP)-resistant cell lines NCI-H446/CDDP and H69/CDDP were also purchased from Shanghai Institute of Cell Biology, Chinese Academy of Science. The cells were also cultured in DMEM medium containing 0.1 mM of cisplatin to maintain the drug resistance in an incubator with 5% CO_2_, at 37°C for conventional culture. The cultured cells were digested and passaged every 2–3 days and the cells at the logarithmic growth phase were used for further experiments. The NCI-H446/CDDP and H69/CDDP cells were divided into four groups: the blank group (without any treatment), tunicamycin group (treated with 5 ug/mL of an ESR inducer tunicamycin), BEZ235 (treated with 64 μM of a inhibitor of PI3K/AKT/mTOR pathway BEZ235; Sigma, USA) group and tunicamycin + BEZ235 group (treated with 5 ug/mL of tunicamycin plus 64 μM of BEZ235) [52].

The article "Activation of endoplasmic reticulum stress promotes autophagy and apoptosis and reverses chemoresistance of human small cell lung cancer cells by inhibiting the PI3K/AKT/mTOR signaling pathway" was retracted in 2019. Reasons: errors in the analysis; false authorship; concerns about the results or conclusions; concerns about a third party's involvement.

### Cell counting Kit-8 (CCK-8) assay

The cells at the logarithmic growth phase were re-suspended in the cell growth liquid. The cell density was adjusted into 1.0 × 10^4^/mL and the cells were mixed evenly to be spread in 96-well plates with 100 μL cell suspension in each well. After the cells were cultured adherent to wall for 24 h, the cell culture medium was discarded. Then 100 μL 5 ug/mL tunicamycin (Sigma-Aldrich Chemical Company, St Louis MO, USA) [53, 54] was added, and 3 repeated wells were arranged. Cells were cultured and observed for 24 h, followed by calculating cells survival rate in each group.

A total of 100 μL of cells culture medium containing tunicamycin (Sigma, USA) at different concentrations of 0 μg/mL, 1 μg/mL, 2 μg/mL, 4 μg/mL, and 8 μg/mL respectively and three repeated wells were arranged. After the cells were cultured for 24, 48 and 72 h, CCK-8 (10 μL, Sigma, USA) solution was added into each well at dark for incubation for 3 h. Culture medium in the 96-well plate was carefully sucked out and DMEM (90 μL) was added into each well at dark. The mixture was shaken using a shaker at dark to be dissolved for 15 min and the dissolved mixture was detected using a micro-plate reader. The optical density (OD) of each well at a 450 nm wavelength was detected. Cell viability under different concentrations of tunicamycin was calculated, that is, the cytotoxicity of cells at different concentrations of tunicamycin and the 50% inhibition (IC50) value was calculated. The concentration and corresponding time were used to conduct the subsequent experiments on chemoresistance.

### Flow cytometry

The supernatant and the adherent cells of another group of drug-treated samples were collected into centrifuge tubes; 2 mL MDC containing medium was added to each well (final concentration: 5 μM); the cells were cultured at an incubator containing 5% CO_2_ at 37°C in the dark for 20 min; the collected supernatant and cells were centrifuged at 2000 rpm for 5 min; the supernatant was discarded, 500 μL MDC containing culture medium was added to each tube (final concentration: 5 μM), the mixture was pipetted and mixed evenly, and the cells were incubated in the dark for 30 min; and the incubated cells were screened over 300 mesh copper grids. The MDC staining fluorescence intensity at an excitation wavelength of 488 nm was detected by the flow cytometry.

The article "Activation of endoplasmic reticulum stress promotes autophagy and apoptosis and reverses chemoresistance of human small cell lung cancer cells by inhibiting the PI3K/AKT/mTOR signaling pathway" was retracted in 2019. Reasons: errors in the analysis; false authorship; concerns about the results or conclusions; concerns about a third party's involvement.

### Flow cytometry after annexin-V/propidium iodide (PI) staining

Cells were digested with ethylene diamine tetraacetic acid (EDTA)-free trypsin (not excessive digestion), the digested cells were collected, and the collected cells were centrifuged at 2000 rpm/min for 5 min, and the centrifuged cells were washed twice with pre-cooled PBS. The washed cells were centrifuged and collected, and the treated cells (1 × 10^6^) were transferred into an Ependorff (EP) tube and 500 μL of bidding buffer was added into each EP tube, and the mixture was mixed evenly. PI (5 μL) and Annexin V (5 μL) (KeyGEN BioTECH, Nanjing, China) were added into each EP tube. After the dyes were added, the cells were incubated in the dark for 10–15 min. The incubated cell suspension was filtered through 400 mesh cell screen to filter off the cell clumps. After filtration, the cells were placed on ice and then detected and analyzed within 30 min using a flow cytometer. AnnexinV^+^PI^−^ indicated early apoptosis and AnnexinV^+^ PI^+^ indicated late apoptotic. Apoptotic rate = early apoptosis rate + late apoptosis rate.

### Western blotting

The cells were collected and the cells adhere to walls were digested by trypsase. After centrifugation, the cells were washed twice with PBS and a right amount of pre-cooled cell lysate was added into the cells. The cell lysis on ice was conducted for 30 min. The lysed cells were centrifuged at 12,000 r/min and 4°C for 20 min. The fully lysed cell liquid was centrifuged at 13,000 rpm, and supernatant was taken and transferred to the EP tube. The supernatant was the extracted total cellular protein. Bicinchoninic acid assay (BCA) protein concentration measuring kit was used to measure the protein concentration, which was adjusted in each group. Protein extracts were quantified, finally 5 × SDS loading buffer was added, and the whole mixture was placed at a high temperature of 95°C to conduct denaturation for 5 min, and the denatured proteins were subjected to SDS-PAGE electrophoresis. The electrophoresed proteins were transferred to a membrane and 5% non-fat dry milk was added into the membrane, and the mixture was sealed overnight at 4°C and washed by tris-buffered saline tween-20 (TBST). Primary antibodies (protein kinase R-like endoplasmic reticulum kinase(PERK): CST, product code: # 5683; eukaryotic initiation factor 2α (eIF2α): CST, product code: # 5432; C/EBP homologous protein (CHOP): CST, product code: # 2895; Beclin1: CST, product code: # 3495; light chain 3 (LC3): CST, product code: # 3868; LC3-I: CST, product code: # 4108; LC3-II: CST, product code: # 2775; p62: CST, product code: # 8025; B-cell lymphoma 2 (Bcl-2): CST, product code: # 2870; Bax: CST, product code: # 5023; procaspase-3: CST, product code: # 9665; PI3K: CST, product code: # 4292; protein kinase B (AKT): CST, product code: # 4691; mammalian target of rapamycin (mTOR): CST, product code: # 2983; phosphorylated-(p-) PI3K: CST, product code: # 4228; p-AKT: CST, product code: # 4060; p-mTOR: CST, product code: # 2971; internal reference glyceraldehyde phosphate dehydrogenase (GAPDH): CST, product code: # 5174) were added, the mixture was incubated overnight. The incubated mixture was washed with TBST, and horseradish peroxidase (HRP) secondary antibodies were added, and the mixture was incubated 37°C for 1 h. The incubated mixture was washed with TBST. HRP electrogenerated chemiluminescence (ECL) was used to develop, the developed films were taken and rinsed with pure water, and the washed films were dried. Scanning was used for recording.

The article "Activation of endoplasmic reticulum stress promotes autophagy and apoptosis and reverses chemoresistance of human small cell lung cancer cells by inhibiting the PI3K/AKT/mTOR signaling pathway" was retracted in 2019. Reasons: errors in the analysis; false authorship; concerns about the results or conclusions; concerns about a third party's involvement.

### Statistical analysis

SPSS13.0 statistical software (SPSS, Inc, Chicago, IL, USA) was used to analyze data. The experiment was repeated three times. Measurement data were expressed as mean ± standard deviation. Differences between groups were analyzed using *t*-test while differences among groups were analyzed using One-way analysis of variance (ANOVA). A *P* < 0.05 indicated significant different and a *P* < 0.01 indicated highly significant different.
